RETRACTED

# The Design and Implementation of Postprocessing for Depth Map on Real-Time Extraction System

**DOI:** 10.1155/2014/363287

**Published:** 2014-06-04

**Authors:** Zhiwei Tang, Bin Li, Huosheng Li, Zheng Xu

**Affiliations:** ^1^Shanghai University, Shanghai 200072, China; ^2^The Third Research Institute of Ministry of Public Security, Shanghai 201204, China; ^3^Tsinghua University, Beijing 100084, China

## Abstract

Depth estimation becomes the key technology to resolve the communications of the stereo vision. We can get the real-time depth map based on hardware, which cannot implement complicated algorithm as software, because there are some restrictions in the hardware structure. Eventually, some wrong stereo matching will inevitably exist in the process of depth estimation by hardware, such as FPGA. In order to solve the problem a postprocessing function is designed in this paper. After matching cost unique test, the both left-right and right-left consistency check solutions are implemented, respectively; then, the cavities in depth maps can be filled by right depth values on the basis of right-left consistency check solution. The results in the experiments have shown that the depth map extraction and postprocessing function can be implemented in real time in the same system; what is more, the quality of the depth maps is satisfactory.

## 1. Introduction 

Real-time stereo vision has been widely used in intelligent smart human-computer interaction, robot navigation, and intelligent surveillance; it maybe becomes an important component in the information of the video structural description [1]. Inspired by human visual process, we can get the stereo vision by calculating the disparity between correspondence points in multiple images captured by corresponding cameras. The stereo vision algorithms are computationally intensive, involving a large number of regular, repetitive operations on large sets of structured data. We know that the algorithms are always implemented by traditional software and that they run on CPU-based platforms, which, using sequential instruction execution mode and fixed control mechanism, will spend a lot of time and cannot satisfy the complete video-rate processing demand. Executing a medium-sized stereo vision algorithm for a single pair of images will consume 5~8 second on a 1 GHz general-purpose microprocessor. This low frame rate results in limited applicability of stereo vision, especially for real-time applications, because quick decisions must be made based on the vision data [2]. We can try some other platforms, for example, FPGA.

The MVD (video + depth) model has become a research hotspot [2] of the stereo video capture in the 3DTV system. The efficiency of depth map extraction affects the whole execution efficiency of the 3DTV system, in the other way; the quality of the depth map also directly determines the effect of rendering, so the extraction efficiency and quality of the depth information are crucial to the 3DTV system.

RETRACTED

The depth information usually can be extracted by some local stereo matching algorithm [3] in some special occasion, in which the depth map was required to be got in real time and FPGA was usually selected as the implementation platform [4]. Because of the characteristics of hardware structure, it cannot realize the complex stereo matching algorithm; unlike the software, on the other hand, local stereo matching algorithm has its own limitation as it cannot get the desired effect when the processed picture contains weak texture, repetitive texture, and noise; mismatching phenomenon was inevitable in the result [5]. According to the above problem, the paper designed the depth map postprocessing function based on depth map real-time extraction system by FPGA that corrects the mismatching point and fills the hole on the initial depth map. As a whole, the depth map postprocessing module is added to the depth information extracting system and the quality of the depth map can be improved obviously.

## 2. Background

Figure 1 shows that a 3DTV construction stereo vision system [6] based on binocular disparity theory and depth estimation codec should include the source video data generation, source data codec, scene reconstruction, and 3D display. Depth map or the 3D information is generated in the transport end and utilized in depth image-based rendering (DIBR) [7] in the receiver end. In this paper we will pay attention to the part of the depth estimation, especially its postprocessing.

By opportunely processing the couple of stereo images captured by two distinct cameras at a distance *b*, called baseline, we can extract depth information. In stereo vision processing, the correspondence search is the main work to solve the stereo matching problem and then furnishing a map of disparity values as a result.

As shown in Figure 2, *Ir* and *Il* in the right and left images, respectively, are the projections of the same point *P* in the real scene, whose position displacement between the corresponding pixels is the disparity. The *z* presents the distance of the point *P* from the stereo camera that can be calculated from the disparity *d* through triangulation computations. We can hypothesize that the focal length of the stereo camera is *f*; taking the baseline *b* into consideration, the depth of the point *P* is *z* and can be calculated by the following formula [8]:

(1) z=b·fd.

RETRACTED

There are mainly two kinds of stereo matching algorithms for calculating the disparity maps, divided into the local and global. The local methods are based on local information around certain positions of pixels, including area based, phase based, and the feature based (matching on features like lines, corners, and edges) methods. Methods such as belief propagation, graph cuts, and dynamic programming are more complex and can be attributed to the global class methods, because they attempt to minimize an energy function computed on the whole image area.

We can contrastively evaluate the quality and performance of the depth map through benchmark images provided with accurate ground truth disparity maps. If the correspondence search is executed along just one dimension of the image area, local methods can be implemented very efficiently; thus, reducing the complexity can be done.

As shown in Figure 2, *Fr* and *Fl* are the two focal points of the right and left cameras, respectively. The above two focal points intersect the left and right images in two specific points *el* and *er* called left and right epipoles. If *Ir*1 is the projection of the generic point *P*1 into the right image, its corresponding point *Il*1 in the left image has to be searched for on the left epipolar line obtained connecting *Il*1 with the left epipole.

At the encoder, a video signal and the corresponding depth map will be encoded and transmitted. From the video and depth information, a stereo pair can be rendered at the decoder, so we can get stereo vision. If the user's head motion is tracked, we can get the head motion parallax viewing and this is an extended function. Efficient compression can be achieved through this way of video plus depth. Per sample depth data can be regarded as a monochromatic, luminance-only video signal, as shown in Figure 3. The depth is restricted to a range between two extremes *Z*_near_ and *Z*_far_, which indicate the minimum and maximum distance of the corresponding 3D point from the camera, respectively. The depth range is linearly quantized with 8 bits; that is, the closest point is associated with the value 255; the most distant point is associated with the value 0. Based on the above description, the depth map can be specified as grey scale image. These grey scale images can be fed into the luminance channel of a video signal and the chrominance can be set to a constant value. The resulting standard video signal can then be processed by any state-of-the-art video codec.

In the project of the European ATTEST [9, 10], the results have shown that depth data can be very efficiently compressed this way. MPEG-2, MPEG-4, H.264/AVC, and so on have been tested; they work well. A course estimate indicates that 10%~20% of the bit rate [11], which is necessary to encode the colour video, is sufficient to encode the depth at good quality. This is due to the specific statistics of depth data, being on average smoother and less structured than colour data.

RETRACTED

Based on these observations, a new backward compatible (with respect to classical DVB) approach for 3DTV was developed in the ATTEST project. It uses layered bit stream syntax. The base layer is a conventional 2D colour video encoded using MPEG-2. This base layer can be processed by any existing MPEG-2 decoder providing backward compatibility. Additionally the bit stream contains an advanced layer carrying the encoded depth information. Advanced systems may access this layer to decode the depth stream and then generate a stereo pair to be displayed stereoscopically by view interpolation.

This concept is highly interesting due to the backward compatibility, compression efficiency, and extended functionality compared to conventional stereo video. Moreover, it does not introduce any specific coding algorithms. It is only necessary to specify high-level syntax that allows a decoder to interpret 2 incoming video streams correctly as colour and depth. Additionally information about depth range needs to be transmitted. Therefore, MPEG specified a corresponding container format “ISO/IEC 23002-3 representation of auxiliary video and supplemental information,” also known as MPEG-3 Part 3, for video plus depth data. Moreover, H.264/AVC contains an option to convey the depth images through its auxiliary picture syntax. Here, the video codec for the color video signal and associated depth video signal are both H.264/AVC. This approach is backwards compatible with any existing deployment of H.264/AVC.

A general problem of the video plus depth format is content creation, that is, the generation of depth information. Cameras that automatically capture per pixel depth with the video are available and are being further enhanced, but the quality of the captured depth fields is currently still limited. Algorithms for depth estimation have been studied extensively in computer vision literature and powerful solutions are available. However, it always remains an estimation that can only be solved up to a residual error probability. Estimation errors influence the quality of rendered views. A fully automatic, accurate, and reliable depth capturing system is still to be developed. User-assisted content generation is an option for specific applications. Even having perfect depth available, artifacts may occur in rendered views due to disocclusion. This effect increases with the distance of the virtual view from the original camera position. Additional occlusion layers (layered depth video as extension of layered depth images) or extension to multiview video plus depth help to minimize these problems at the cost of increased data rate and complexity.

RETRACTED

## 3. The Real-Time Depth Map Extracting System

Stereo vision refers to the issue of determining the 3D structure of a scene from two or more images taken from distinct viewpoints. In the case of a binocular stereo, the depth information for the scene is determined by searching the corresponding pairs for each pixel within the image. Since this search method is based on a pixel-by-pixel comparison, which consumes much computational power, most stereo matching algorithms have assumptions about the camera calibration and epipolar geometry [12].

An image transformation, known as rectification, is applied in order to obtain a pair of rectified images from the original images as in (2). In the equations, (*x*, *y*) and (*x*′′, *y*′′) are the coordinates of a pixel in the original images and the rectified images, respectively. To avoid problems such as reference duplication, reverse mapping is used with interpolation. Once the image pair is rectified, 1D searching with the corresponding line is sufficient to evaluate the disparity [13]. Consider

(2) $$\begin{array}{c} \left[\begin{array}{c} x_{l}^{\prime }\\ y_{l}^{\prime }\\ z_{l}^{\prime } \end{array}\right]=H_{l}^{-1}\left[\begin{array}{c} x_{l}^{\prime \prime }\\ y_{l}^{\prime \prime }\\ 1 \end{array}\right],\\ \left[\begin{array}{c} x_{r}^{\prime }\\ y_{r}^{\prime }\\ z_{r}^{\prime } \end{array}\right]=H_{r}^{-1}\left[\begin{array}{c} x_{r}^{\prime \prime }\\ y_{r}^{\prime \prime }\\ 1 \end{array}\right],\\ \left[\begin{array}{c} x_{l}\\ y_{l} \end{array}\right]=\left[\begin{array}{c} \frac{x_{l}^{\prime }}{z_{l}^{\prime }}\\ \frac{y_{l}^{\prime }}{z_{l}^{\prime }} \end{array}\right],\\ \left[\begin{array}{c} x_{r}\\ y_{r} \end{array}\right]=\left[\begin{array}{c} \frac{x_{r}^{\prime }}{z_{r}^{\prime }}\\ \frac{y_{r}^{\prime }}{z_{r}^{\prime }} \end{array}\right]. \end{array}$$

After rectification, stereo matching (given a pixel in one image, find the corresponding pixel in the other image) is applied to solve the correspondence problem. Since pixels with the same intensity value can appear many times within the image, a group of pixels, called windows, is used to compare the corresponding points. Several stereo vision algorithms were introduced based on different correspondence methods, local and global. The local method includes block matching, feature matching, and gradient-based optimization, while the global method includes dynamic programming, graph cuts, and belief propagation. Because we can restrict the searching range of stereo matching to one dimension, local methods can be very efficient compared with global methods. Moreover, even though local methods experience difficulties in locally ambiguous regions, they provide acceptable depth information for the scene with the aid of accurate calibration [14]. For this reason, we employed the local stereo method as the cost function of the proposed system. In particular, we used census-based correlation because of its robustness to the random noise within a window and its bit-oriented cost computation.

RETRACTED

The census transform maps the window surrounding the pixel *p* to a bit vector representing the local information about the pixel *p* and its neighboring pixels. If the intensity value of a neighboring pixel is less than the intensity value of pixel *p*, then the corresponding bit is set to 1; otherwise, it is set to 0. The dissimilarity between two bit strings can be measured through the hamming distance, which determines the number of bits that differ between these two bit strings. To compute the correspondence, the sum of these hamming distances over the correlation window is calculated in (3), where *I*_1_′ and *I*_2_′ represent the census transform of template window *I*_1_ and candidate window *I*_2_ [15]. Consider

(3) $$\begin{array}{c} \underset{\left(u,v\right)\in W}{\sum }\text{Ham}\;\min\;g(I_{1}^{\prime }\left(u,v\right),I_{2}^{\prime }\left(x+u,y+v\right)). \end{array}$$

The results for stereo matching provide a disparity, which indicates the distance between the two corresponding points. For all possibilities, the disparity should be computed and evaluated at every pixel within the searching range. However, reliable disparity estimations cannot be calculated on surfaces with no texture or repetitive texture when utilizing a local stereo method [16]. In this case, the disparities at multiple locations within the image may point to the same location in the other image despite each location within one image being assigned, at most, one disparity. This unique test method tracks the three smallest matching results *v*_1_, *v*_2_, and *v*_3_, instead of seeking only the minimum. The pixel has a unique minimum if the minimum, *v*_1_, lies between *v*_2_ and *v*_3_, as in (4), where *N* is an experimental parameter. Usually, the value of *N* lies between 1.25 and 1.5; we used a value of 1.33 in all our experiments. Consider

(4) $$\begin{array}{c} v_{2}>Nv_{1},\;\;v_{3}>Nv_{1}. \end{array}$$

As shown in Figure 4, it is the structure schematic diagram of the real-time depth map extracting system based FPGA, which is mainly used to obtain the depth map of the dual view or multiview video in the 3DTV system. (a) is the binocular SDI high-definition cameras; (b) is the FPGA development platform that is used to implement the algorithm; (c) is the encoder of the 3DTV system, which is designed to encode the real-time depth information; (e) is the FPGA chip for the SDI protocol parsing, stereo matching, detection of the matching unique, left-right consistency detection, filling the hole in the depth map, and so on.

RETRACTED

After SDI protocol parsing, the depth map can be extracted. As shown in Figure 4, (A) is the depth extracting module, including the census regional transformation, matching cost accumulation, WTA [7, 17, 18], and optimal choice. (B) is mismatch detection and postprocessing module, containing matching unique detection, left-right consistency detection, and so on.

## 4. The Implementation of the Postprocessing for the Depth Map

There are some error matching points introduced by match methods and freedom noises. In order to improve the quality of depth map, approaches should be taken. The manual edge map and manual depth map have been taken to correct the object edges and other errors. However, the manual processing introduces much more complicated algorithm, for example, edge detection, segmentation, graph cut, and so on. Depth map cannot be generated automatically. It will result in increasing hardware design complexity and increasing the circuit scale. Here we find that discrete wavelet transform (DWT) has low-pass filter and high-pass filter operation, and it is fit for hardware design during optimizing the depth map. DWT is a multiresolution decomposition processing. Shape-adaptive discrete wavelet transforms (SA-DWT) is an improved algorithm. With the regular algorithm, images can be separated into skeleton and details. The other advantage is the decomposition, and the reconstruction process can be considered as a mathematical reverse operation. It is helpful for the reuse of hardware sources.

In the depth map real-time extraction system, after getting the parallax value each pixel corresponds to, in order to improve the quality of depth map, there shall be a postprocessing for the depth map. In this section we focus on designing and implementation process of the depth map postprocessing.

### 4.1. Detection of the Matching Unique

In the stereo matching process, we can get the parallax value by WTA algorithm after matching cost measure criterion is established. There may be some matching point, whose match cost is close to the minimum matching value, leading to the corresponding Parallax being unstable [19]. We can overcome this problem by detecting the minimum match cost. The concrete expression is shown in the following formula:

(5) $$\begin{array}{c} \frac{\text{va}{\text{l}}_{0}}{\text{va}{\text{l}}_{1}}>\text{th}. \end{array}$$

th is the default threshold which can be set according to the experience and the general value is in the scope of 1.2~1.5. The th will be set as 1.33 in our design. val_0_ is the second lowest value of all parallax in the search scope and val_1_ is the lowest value of all. When the value meets the above formula and the difference between the val_0_ and val_1_ is greater than a specific value, we choose the val_0_ as the accurate value and make the corresponding point in the picture as the stable point, and that means parallax uniqueness results satisfy matching detection. If formula (5) is not observed, the corresponding point will be divided into the unstable points for processing.

RETRACTED

The direct implementation of the decimal and division calculations are quite complex by hardware; we can achieve the same effect by adder and comparator instead of the complicated operation. The specific RTL block diagram is shown in Figure 5.* COMP4X*,* COMP3X* are the val_1_, val_0_, respectively, in formula (5). For* COMP4X*, shift it to the left by 2 bits, shift the* COMP3X* to the left by 1 bit, and then add its original value. Comparing the* COMP4X* with* COMP3X*, we can get the result* COMPOUT*; if the value of the* COMPOUT* is 1, it means that formula (5) will be workable when th is set to 1.33.

### 4.2. Left-Right Consistency Check

The left-right consistency check [20] is based on the reversible match hypothesis, whose specific content is that: taking the left view as reference, find the matching point as reference point in the right view. In turn, we can search the matching point in the left view. This detection method is also known as cross test. In all matching points, which are obtained based on the benchmark of left-right view, only the points whose left and right points matched each other are the effective matching point-pair. We can get high detection rate for the shade area in the picture by this method. Consistency criterion can be represented as follows:

(6) $$\begin{array}{c} d_{\text{LR}}\left(x,y\right)=-d_{\text{RL}}\left(x+d_{\text{LR}}\left(x,y\right),y\right). \end{array}$$

The *d*_LR_, *d*_RL_ are the parallax base on the left and right view picture, respectively. Mark the points that do not satisfy the hypothesis as the unreliable points. In consideration of the lack of the subpixel accuracy, the deviation of the parallax base on the left-right view is allowed to range from 0 to a pixel in the process of the hardware implementation or the corresponding parallax will be set as invalid value.

RETRACTED

It is worth noting that the parallax referenced against the right view will lag behind the right original view for 64-clock period after stereo matching. Because the pixels of the same picture are left to the right view and right to the left view, in order to get the parallax of the pixel from the right view, we must hold clocks within the scope of a parallax (the number of the clocks within the scope of a parallax is set as 64 in the test system) to wait the corresponding pixels in the left view and then the stereo matching can be implemented under the same clock.

In order to get the parallax of the left view by the left-right consistency model, the 64-clock delay model will be added before the sequential operation process in Figure 6 can explain why.

After adding the time delay model, the left and right parallaxes that are put into left-right consistency check model will be in synchronous alignment. The pixel in the right view will be got earlier than that in the left view and the time interval ranges from 1 to 64 clocks. The parallax of the right view can be stored in 64 registers; when the parallax value of the left is *n*, we can check if the parallax of a specific pixel conforms with the left-right consistency or not by judging the time in the *n*th register of the right view if it ranges within the scope of ±1.

The process of the above storage and the comparing are shown in Figure 6. There is an example of the left-right consistency check of three possible parallaxes in a pixel in that figure. At any given time *T*0 in the horizontal axis, there may be three possible parallaxes for a pixel in the left view: when the value is 5, store the right view parallax and then the value in register *R*5 is 5; in the same way, for the two other possible parallaxes, the values of the *R*10 and the *R*32 will be 10 and 32, respectively. The above three kinds of hypotheses satisfy the left-right consistency check; if the value of the register *Rn* is out of the range from *n* − 1 to *n* + 1, it means that the parallax of the left view cannot meet the consistency check.

In fact, if the left view does not delay for 64 clocks, in other words, the matching result of the left and right view will be input to the left-right consistency check model directly. As shown in Figure 7, the scheme of comparison between the previous parallax of right view and the current parallax of the left view is no longer applicable. The left-right consistency checking can only be implemented as in Figure 7.

In the parallax of the right view, if the value is 30, the corresponding parallax in the time *T*0–64 is *a* in the right view. Normally, if the point *a* in the left view shifts to the right by 30 pixels, its corresponding parallax will be 30; that value will be stored 35 times by shift registers and the *R*35 = 30 in *T*0. Similarly for the second and the third hypotheses, the value of *R*10, *R*3 should be 55 and 62. Those three examples conform to the left-right consistency. If the register *Rn* ≠ (64 + 1 − *n* ± 1), the corresponding parallax in the right view does not meet the consistency.

RETRACTED

### 4.3. File the Hole of the Depth Map

The left-right consistency checking can filter out a lot of false matching points, especially, some mismatching point caused by shading. We can improve the accuracy and robustness of depth extracting, but inevitably this leads to a large hole appearing in the covered area in the depth picture. The depth, in which some cavities exist at the shelter, for virtual visual mapping, will inevitably lead to crack of edges.

Because the covered pixels miss effective match information, the content in the hole is the background, so we can make use of the information of the background pixel to fill the hole [20–23].

In Section 2, the paper provides two structures about left-right consistency checking. We can get the depth map by the left view in the first structure, in which there are some holes in the right, and the corresponding background pixels are right to the holes. We know that the pixel in the video stream will appear from left to right in turn, and the right pixel in the picture is the unknown data for the left. We can only store the known date to fill the hole and the reverse is false [20]. So the right background depth cannot be used to fill the hole. In the second structure, we can store the depth value, whose corresponding pixels pass the left-right consistency checking and fill the hole directly.

## 5. Experimental Results and Analysis

This section will analyze the depth map extraction and postprocessing system from two aspects: the depth map effect and the hardware resource occupancy.

### 5.1. The Result of the Depth Map Extraction

The depth map is shown in Figure 8, and the resolution of the original picture is 1920 by 1080.

The system uses stereo matching algorithm based on nonparametric region transform to achieve stereo matching [19]; it can be seen from Figure 8; although the effect of the local stereo matching algorithm is not as good as global stereo matching, the chairs, flooring, and the remarkable objects in indoor environments have the better quality depth map, and the nonparametric transform stereo matching has better robustness for noise and uneven illumination. Overall, the depth map extraction and the corresponding postprocessing mode can be real-time implemented and the system has practical application significance.

RETRACTED

### 5.2. The Occupancy of Resource

The main chip in experiment system is Altera Arria II GX260; there are a lot of resources for storage and high-speed parallel computing in the chip. After adding depth extraction and postprocessing algorithm, in conjunction with the external SDI resolved, DDR2 cache, PCIE transmission module, and its main internal resources are shown in Table 1.

As can be seen from the table the resource in chip can be reasonably utilized. Although the depth chart of the high-resolution video processing requires more hardware resources, the occupancy rate of the resources can be effectively kept within a reasonable range in the premise of guaranteeing real-time operating by rational design, flexible use of the area, and speed swap ideas.

## Figures and Tables

**Figure 1:** 3DTV system.

**Figure 2:** Epipolar geometry.

**Figure 3:** The 3DTV data representation using video plus depth.

**Figure 4:** Depth map real-time extraction system structure diagram.

**Figure 5:** The RTL schematic of comparison module in the unique matching detection.

**Figure 6:** The sequential process about getting the parallax of the left view.

**Figure 7:** The sequential process about getting the parallax of the right view.

**Figure 8:** The extraction of the depth map.

**Table 1:** The occupancy of FPGA resource.

Item	Content		Remark
FPGA type	EP2AGX260EF29C4		Altera (Arria II GX260)
FPGA resource	Total pins	206/432	48%
	Total block memory bits	3004880/8755200	34%
	Total DSP block 18-bit elements	0/736	0%
	Total GXB receiver channel PCS	8/12	67%
	Total GXB receiver channel PMA	8/12	67%
	Total GXB transmitter channel PCS	8/12	67%
	Total GXB transmitter channel PMA	8/12	67%
	Total PLLs	2/6	33%
	Total DLLs	1/2	50%
	PCIE hard IP	1/1	100%
	Logic utilization	34%	
	Combinational ALUTs	35717/205200	17%
	Memory ALUTs	24/102600	<1%
	Dedicated logic registers	60363/205200	29%
	Total registers	60799	
